# Yap-Hippo Signaling Activates Mitochondrial Protection and Sustains Breast Cancer Viability under Hypoxic Stress

This article has been retracted.

**DOI:** 10.1155/2021/5212721

**Published:** 2021-09-13

**Authors:** Chen Shi, Siyuan Zhang, Changkuo Guo, Jian Tie

**Affiliations:** Department of Radiation Oncology, Key Laboratory of Carcinogenesis and Translational Research (Ministry of Education/Beijing), Peking University Cancer Hospital and Institute, Beijing 100142, China

## Abstract

Yes-associated protein (Yap) is a transcriptional regulator that upregulates oncogenes and downregulates tumor repressor genes. In this study, we analyzed protein expression, RNA transcription, and signaling pathways to determine the function and mechanism of Yap in breast cancer survival during hypoxic stress. Yap transcription was drastically upregulated by hypoxia in a time-dependent manner. siRNA-mediated Yap knockdown attenuated breast cancer viability and impaired cell proliferation under hypoxic conditions. Yap knockdown induced mitochondrial stress, including mitochondrial membrane potential reduction, mitochondrial oxidative stress, and ATP exhaustion after exposure to hypoxia. It also repressed mitochondrial protective systems, including mitophagy and mitochondrial fusion upon exposure to hypoxia. Finally, our data showed that Yap knockdown suppresses MCF-7 cell migration by inhibiting F-actin transcription and promoting lamellipodium degradation under hypoxic stress. Taken together, Yap maintenance of mitochondrial function and activation of F-actin/lamellipodium signaling is required for breast cancer survival, migration, and proliferation under hypoxic stress.

## 1. Introduction

Breast cancer is the most commonly diagnosed cancer in women, with an estimated 268,600 newly diagnosed women with invasive disease in 2019 in the United States [1]. Approximately 42,000 women are expected to die in the US from breast cancer each year, making it as the second-leading cause of cancer-related death among US women after lung cancer [2]. Although breast cancer generally has been identified as a single disease, there are up to 21 distinct histological subtypes and at least four different molecular subtypes [3]. Most cases (80%) are invasive, or infiltrating, and while black and white women in the US are diagnosed at roughly the same rate, the relative survival rate was 83% for black women and 92% for white women [4].

Yes-associated protein (Yap) was originally reported as a transcriptional regulator that upregulates the transcription of oncogenes and reduces the levels of tumor suppressors. Under physiological conditions, Yap is primarily found unphosphorylated in the cytoplasm. After stimulation by hypoxia and inflammation, Yap is phosphorylated at Ser127 [5] and translocates into the nucleus, where it regulates gene expression related to tumor development with the help of transcriptional coactivators with a PDZ-binding motif (TAZ) [6]. Accordingly, several researchers have proposed that Yap is a critical factor in cancer genesis and development. Our previous study [7] revealed a link between Yap activation and hepatocellular carcinoma invasion. We found that Yap inhibited JNK phosphorylation and thus sustained the levels of mitochondria-generated ATP, favoring cancer migration and mobilization. In addition to liver cancer, abundant expression of Yap modulates the activity of macrophage stimulating 4 (MST4) kinase and is also associated with gastric tumorigenesis [6]. The metabolic reprogramming in neural crest is also controlled by Yap signaling [8]. In colorectal cancer, the level of intracellular total Yap rather than its phosphorylation status has been used as a prognostic biomarker [9]. In breast cancer, recent studies have shown that Yap activates the ubiquitin ligase RNF187 and is a potential target for the treatment of triple negative breast cancer [10]. Moreover, anti-HER2 treatment resistance in breast cancer seems to be also associated with Yap.

Tumor hypoxia occurs when tumor cells rapidly outgrow their blood supply, reducing oxygen concentration in the tumor. Although excessive hypoxia would impair cancer metabolism and thus induce cancer cell death or proliferation arrest, the presence of hypoxic regions is one of the negative independent prognostic factors for human cancer [11, 12]. Under hypoxic conditions, hypoxia-induced factor 1 (HIF1) is activated to upregulate the transcription of genes that are involved in angiogenesis, cell survival, and glucose metabolism. For example, overexpression of HIF1 promotes cancer metastasis [13]. HIF-1 promotes the Warburg effect, the tumor-related metabolic switch, which helps cancer cells create energy largely by disintegration of glucose in a nonoxidative manner rather than typical oxidative phosphorylation. Due to decreased oxygen delivery, VEGF expression is upregulated by HIF1 activation and contributes to the formation of blood vessels [14]. HIF1 appears to play a critical role in preventing cell death and promoting cancer proliferation through upregulation of the transcription and expression of cell-cycle-related proteins such as Cyclin D and p21 [15]. Notably, the relationship between Yap and HIF1 has been reported in gastric cancer [16], liver cancer [17], and pancreatic cancer [18], but not in breast cancer. Therefore, the aim of our study was to explore the role of Yap in breast cancer survival and determine whether Yap affects breast cancer cell death through HIF1 under a hypoxic environment.

## 2. Materials and Methods

### 2.1. Cell Culture and Treatment

Human breast cancer cell line MCF-7 was purchased from the American Type Culture Collection (ATCC, Manassas, VA, USA) [19]. We cultured cells in RPMI 1640 medium supplemented with 10% FBS (ExCell Bio, China), 100 mg/ml streptomycin, and 100 U/ml penicillin (Gibco; Thermo Fisher Scientific, Inc., Grand Island, NY) in an incubator at 37°C with 5% CO_2_ [20]. Hypoxia treatment was induced in the hypoxic incubator at 37°C with 1% O_2_.

### 2.2. Quantitative Real-Time- (qRT-) PCR

Reverse transcription was performed using qScript microRNA cDNA Synthesis Kit (Quanta). PCR was performed using an ABI PRISM Sequence Detector System 7500 (Applied Biosystems) with SYBR Green (Quanta) as the fluorescent dye and ROX (Quanta) as the passive reference dye [21]. The cycle number at which the reaction crossed an arbitrarily-placed threshold (CT) was determined for each gene, and the relative amount of each gene to 18S rRNA was used to quantify cellular RNA [22].

### 2.3. Western Blot

Western blotting was conducted with minor modifications. Briefly, cells infected with siRNA were lysed in ice-cold lysis buffer (50 mmol/L Tris-HCl [pH 8.0], 150 mmol/L NaCl, 0.1% Triton X-100, 10 mmol/L EDTA, complete protease inhibitor (Roche), and 20 mmol/L N-ethylmaleimide). For Western blot analysis, approximately 50 *μ*g of protein from each sample was separated by SDS-PAGE and transferred to PVDF membranes (Schleicher & Schuell) [23]. The membranes were blocked with 5% non-fat milk and then incubated with primary antibodies at 4°C overnight. The membranes were incubated with secondary antibodies conjugated to horseradish peroxidase (Jackson ImmunoResearch) and then developed with a chemiluminescent substrate (Perkin Elmer) [24].

### 2.4. Immunofluorescence and Confocal Microscopy

Cells were collected and fixed with 4% paraformaldehyde for 30 minutes at room temperature. Prior to staining, fixed vessels were rinsed with PBS, permeabilized with PBST (PBS with 0.1% Triton X-100) for 10 minutes, and then blocked for nonspecific binding using 5% goat serum for 2 hours at 4°C on a rocker plate [25]. Once blocked, samples were incubated overnight with primary antibodies in PBS [26]. Images were captured using an inverted confocal fluorescence microscope Olympus IX81 with a Hamamatsu C11440 ORCAFlash4.0 digital camera [27].

### 2.5. Mitochondrial Respiration Assays

Respiration was assessed in isolated mitochondria by measuring O_2_ consumption using an Oroboros Oxygraph (Oroboros Instruments, Innsbruck, Austria) [28]. Standardized instrumental and chemical calibrations were performed to correct for backdiffusion of O_2_ into the chamber from leakage, consumption by the chemical medium and sensor consumption [29]. Measurements were taken from 50 *μ*g of mitochondria or 120,000 cells in suspension (2 mL) gently agitated at 37°C. State 2 respiration (mito only) was assessed with the addition of glutamate (10 mM), malate (2 mM), and succinate (10 mM) as the complex I and II substrates, and then State 3 respiration (mito only) was assessed by the addition of ADP (0.5 mM) [30]. State 4 (leak) respiration was assessed with the complex V inhibitor oligomycin (2 *μ*g/mL). Respiration due to reactive oxygen species formation was assessed with Antimycin A (2.5 *μ*m) [31]. O_2_ flux was measured by Datlab2 software (Oroboros Instruments, Innsbruck, Austria), capable of converting nonlinear changes in the negative time derivative of the oxygen concentration signal [32].

Mitochondrial respiration was also assessed in plated cells by measuring O_2_ consumption using the Seahorse XF24 e Analyzer. Cells were grown on a plastic 24-well plate, cultured with Claycomb media and allowed to grow to confluence [33]. Before experimentation, cells were washed with supplemented XF assay media (Seahorse Bioscience, North Billerica, MA) and allowed to equilibrate for 1 h. ATP production, maximal respiration, and nonmitochondrial respiration were assessed by treating cells with oligomycin (1 *μ*m), FCCP (1 *μ*m), and a rotenone (1 *μ*m)/antimycin (1 *μ*m) mixture, respectively [32].

### 2.6. Mitochondrial Membrane Potential/ROS Assessment

Cells were loaded in 96 well plates and then stained with 5 *μ*m MitoSox for 10 min to quantify ROS and 10 nm TMRM for 30 min to quantify changes in mitochondrial membrane potential [34]. Cells were imaged in a widefield fluorescence microscope (ImageXpress Micro, Molecular Devices, Sunnyvale, CA), and changes in intensity means were quantified using Imaris software [35].

### 2.7. Mitochondrial Isolation

Mitochondria were isolated from cells by first detaching cells with 0.05% Trypsin/EDTA for 10 min, washing with Claycomb media and resuspending cells in a minimal volume of isolation buffer. Cells were then lysed by passing through a 27-gauge syringe (15 strokes) [36]. Cell lysates were centrifuged at 500 ×g for 10 min, and the resulting supernatants were centrifuged at 10,000 ×g for 15 min. The mitochondrial pellet was washed once with isolation buffer and the final pellet resuspended in a minimal volume of isolation buffer and kept on ice for functional assays [37]. If samples were used for Western blot, mitochondria were solubilized in isolation buffer containing 1% Triton X and stored at −80°C. Purity of mitochondrial fractions is confirmed by the absence of the cytosolic protein enolase [38].

### 2.8. Generation of Yap Knockout Cell Line

siRNA against Yap was purchased from Addgene. Cells (1 × 10^5^ cells) were plated in a 24-well plate and transfected with siRNA. Forty-eight hours after transfection, FACS (BD FACSAria TM II, BD) was performed to isolate GFP-positive cells [39]. Following isolation, cells were plated in a 96-well plate by limiting dilution for a single-cell cloning. Western blots were used to validate the knockdown efficiency of Yap siRNA [40].

### 2.9. Statistical Analysis

All experiments are presented as mean ± SEM. Statistical analysis was performed using Prism 6 (GraphPad) or SPSS (IBM). Shapiro–Wilk test was used for normality test. Statistical significance was determined by either unpaired *t*-test, one-way ANOVA, or two-way ANOVA followed by Tukey multiple comparison test. If the normality assumption was violated, nonparametric tests were conducted. *p* < 0.05 denotes statistical significance.

## 3. Results

### 3.1. Yap Knockdown Induces Breast Cancer Cell Death and Proliferation Arrest under Hypoxia

After exposure to hypoxic stress, the viability of MCF-7 cells was significantly reduced in a time-dependent manner (Figure 1(a)), suggesting that prolonged hypoxia may cause MCF-7 death. This hypothesis was validated by analyzing TUNEL staining and caspase-3 activity. As shown in Figure 1(b), compared to the control group, the number of TUNEL-positive cells was progressively increased in response to hypoxia treatment, an effect that was followed by an increase in the activity of caspase-3 *in vitro* (Figure 1(c)). These results indicate that excessive hypoxia is a proapoptotic signal for MCF-7 cells *in vitro*. To analyze the role of Yap in hypoxia-related cell damage, siRNA against Yap was transfected into MCF-7 cells as we previously described [7]. Knockdown efficiency was confirmed through qPCR (Figure 1(d)). Then, cell death was analyzed through MTT assay and TUNEL staining. As shown in Figure 1(a), baseline knockdown of Yap had no influence on cell viability but significantly augmented hypoxia-mediated cell death. Similar results were also observed using TUNEL staining (Figure 1(b)), indicating that hypoxia-induced breast cancer cell damage may be amplified due to Yap deficiency.

CCK-8 assay was used to analyze MCF-7 growth under hypoxic stress. As shown in Figure 1(e), compared to the control group, hypoxia slightly reduced the proliferation rate in MCF-7, and this effect could be further augmented by Yap knockdown. The transcription levels of VEGF and *p*21 were moderately downregulated after exposure to hypoxic stress, while Yap knockdown further reduced the levels of VEGF and *p*21 (Figures 1(f) and 1(g)), suggesting that breast cancer cell proliferation is negatively affected by hypoxia and further reduced by Yap deficiency. Notably, since hypoxia for 24 hours caused a statistically significant reduction in MCF-7 viability (Figure 1(a)) and proliferation (Figure 1(e)), 24-hour hypoxia was used in the following experiments.

### 3.2. Yap Knockdown Reduces Mitochondrial Function in Hypoxia-Treated Breast Cancer

Our previous studies [7] showed that mitochondria function downstream of Yap in liver cancer. Loss of Yap induced a decline in mitochondrial ATP production and thus caused intracellular calcium overload, resulting into cancer cell mobilization impairment. Based on these studies [7], we questioned whether mitochondrial dysfunction also occurred downstream as a result of Yap knockdown. Mitochondrial ATP production was reduced slightly by hypoxia and largely by Yap knockdown (Figure 2(a)). Intracellular ATP levels are determined by mitochondrial membrane potential, which converts chemical potential energy to kinetic energy [41, 42]; the latter is used by mitochondria to generate ATP. After exposure to hypoxia, mitochondrial membrane potential was reduced (Figures 2(b) and 2(c)), and this action was further augmented in Yap-knocked down MCF-7 cells, suggesting that Yap is required to sustain mitochondrial potential under hypoxia stimulus. Furthermore, due to a loss of mitochondrial potential, the levels of mitochondrial ROS were also increased under hypoxia, while Yap knockdown multiplied ROS formation (Figures 2(d) and 2(e)).

In addition to mitochondrial dysfunction, we also found that the mitochondrial autophagy system, termed mitophagy, was enhanced during the period of hypoxia (Figure 2(f)), which is in accordance with previous studies [43, 44]. Interestingly, without Yap, mitophagy was significantly reduced, consistent with our previous findings [7], reconfirming that Yap is an activator of mitophagy during hypoxia that enhances mitochondrial self-repair. Additionally, the mitochondrial fusion system attenuates mitochondrial damage through generation of a long, shared electrochemical potential within the mitochondrial network [45, 46]. Mitochondrial fusion also equilibrates mitochondrial proteins, lipids, metabolites, and mtDNA, which is thought to alleviate the local stress response and restore mitochondrial homeostasis [47, 48]. Although mitochondrial fusion parameters were unregulated by hypoxia (Figures 2(g) and 2(h)), Yap knockdown inhibited the activity of mitochondrial fusion in MCF-7 cells.

### 3.3. Yap Activates HIF1 under Hypoxia and Maintains Mitochondrial Homeostasis

To explain the regulatory role played by Yap in mitochondrial homeostasis under hypoxia, we focused on HIF1, which has been identified as a key transcriptional factor activated by hypoxia and contributes to transcription of protective genes [49]. Firstly, we found that the transcription of HIF1 was rapidly increased in response to hypoxia treatment, whereas this trend was reversed by Yap knockdown, suggesting that HIF1 activation requires Yap under hypoxia condition (Figure 3(a)), which is in accordance with the previous studies [50]. This finding was further supported via Figure 3(b). Compared to the control group, HIF expression was augmented by hypoxia, as evidenced by abundant expression of HIF1 in the cytoplasm. However, in MCF-7 cells transfected with Yap siRNA, the levels of intracellular HIF1 were apparently downregulated (Figure 3(b)). These data indicate that hypoxia activates HIF1 through Yap.

To understand whether HIF1 is involved in Yap-related mitochondrial dysfunction, HIF1 adenovirus was transfected into Yap-knockdown cells. Then, mitochondrial function and cell viability were measured again. As shown in Figure 3(c), compared to the control group, intracellular ATP generation was reduced in response to Yap knockdown, and this effect could be attenuated by HIF1 overexpression. Additionally, Yap deletion-mediated ROS overproduction was ameliorated by HIF1 overexpression (Figure 3(d)), reconfirming that HIF1 may function downstream of Yap and sustain mitochondrial homeostasis in MCF-7 cells.

### 3.4. Overexpression of HIF1 Abolishes Yap Knockdown-Mediated Breast Cancer Death and Proliferation Arrest

Next, we explored whether HIF1 overexpression attenuates Yap knockdown-induced breast cancer cell death and proliferation arrest. As shown in Figure 4(a), compared to the control group, Yap knockdown augmented hypoxia-initiated cell death, as evidenced by MTT assay, whereas overexpression of HIF1 maintained MCF-7 cell viability. Similar to these results, TUNEL assay demonstrated that the number of apoptotic cells was increased by Yap knockdown; this effect could be abolished by HIF1 overexpression (Figure 4(b)). In addition to cell death, CCK-8 assay also illustrated that the proliferative capacity of MCF-7 cells was impaired by Yap knockdown, whereas HIF1 overexpression could sustain cancer cell proliferation (Figure 4(c)). This finding was also supported by qPCR for the analysis of cell-cycle-related genes. As shown in Figures 4(d) and 4(e), compared to the control group, the transcription levels of VEGF and *p*21 were reduced by hypoxia, whereas this action could be abolished by HIF1 overexpression.

### 3.5. F-Actin/Lamellipodium Signaling Pathway Is Impaired by Yap Knockdown under Hypoxia

In addition to cancer cell survival and proliferation, invasion is vital for cancer development and progression. Our previous study [7] reported that F-actin and lamellipodium are vital for cancer mobilization. At the molecular level, F-actin multimerizes at the membrane and then forms the lamellipodium, which induces cellular deformation and migration [51]. In this study, immunofluorescence was used to observe alterations in the lamellipodium. As shown in Figures 5(a)–5(c), compared to the control group, the number and length of lamellipodia were significantly reduced in response to hypoxia. After knockdown of Yap, the number and length of lamellipodia further decreased; these effects could be reversed by HIF1 overexpression. Lamellipodium degradation may be a result of F-actin downregulation [52]. Therefore, qPCR was used to analyze the alterations of F-actin. As shown in Figure 5(d), compared to the control group, F-actin transcription was inhibited by hypoxia, and this effect was augmented by Yap deletion. Interestingly, HIF1 overexpression restored F-actin transcription in MCF-7 cells under hypoxia treatment. F-actin downregulation and lamellipodium degradation may impair cancer cell migration [53]. Thus, transwell assay was used to analyze the migratory response of MCF-7 in response to hypoxia and/or Yap knockdown. As shown in Figure 5(e), compared to the control group, the number of migrating MCF-7 cells was reduced after exposure to hypoxic stimulus. Although Yap knockdown further reduced the migratory response in hypoxia-treated MCF-7 cells, HIF1 overexpression could normalize MCF-7 mobility. Overall, this result indicates that Yap knockdown weakens breast cancer mobilization through inhibiting the F-actin/lamellipodium signaling pathway in a manner dependent on HIF1.

## 4. Discussion

In this study, we found that Yap expression is increased in MCF-7 breast cancer cells under hypoxia stimulus. Higher levels of Yap contribute to the survival, proliferation, and migration of MCF-7 breast cancer cells by activating HIF1. Loss of Yap activated apoptosis and limited proliferation in MCF-7 cells through induction of mitochondrial dysfunction. Yap knockdown also blunted the F-actin/lamellipodium signaling pathway, thereby attenuating the MCF-7 migratory response. Mechanistically, Yap knockdown dissipated mitochondrial membrane potential, resulting in ATP undersupply and ROS overproduction. Moreover, Yap knockdown also impaired mitophagy and mitochondrial fusion through an undefined mechanism. Moderately damaged mitochondria fail to produce ATP for cell metabolism and mobilization, whereas excessively injured mitochondria are a trigger for cellular apoptosis. To the best of our knowledge, this is the first study to identify Yap as the master of breast cancer survival through protection of mitochondrial function in the setting of hypoxic stress. This finding defines Yap and its downstream effector, HIF1, as potential targets to prevent breast cancer growth and invasion.

Yap activation plays an important role in decreasing the immune system response [54] and accelerating cancer cell type transition [55]. Tumor cell senescence or reduced stemness is also associated with a drop in the expression of Yap [56]. Interestingly, chemotherapy or radiotherapy resistance mechanisms in prostate cancer [57], gastric cancer [58], bone pediatric cancer [59], and breast cancer [60] are linked to Yap activation or overexpression. We found that hypoxic stress was a critical factor that induces Yap transcription and activation in a time-dependent manner. Considering the tumor-promoting property of Yap, increased levels of Yap may offset the adverse impacts induced by hypoxia, such as apoptosis, migration inhibition, and proliferation arrest. In our study, we found that Yap was required for MCF-7 cell survival and proliferation under hypoxic conditions since knockdown of Yap augmented hypoxia-induced apoptosis [61].

Mechanistically, we found that Yap deficiency was associated with mitochondrial dysfunction including mitochondrial membrane potential reduction, mitochondrial metabolic impairment, and oxidative stress injury. In addition, mitochondrial protective mechanisms such as mitophagy and fusion were also inhibited by Yap knockdown. Our previous studies [7] showed that Yap deletion reduces mitochondrial ATP production and thus impairs liver cancer migration, which is highly dependent on intracellular energy supply. In glioblastoma A172 cells, the loss of Yap prevents the activation of AMPK, a sensor of cellular ATP status [62, 63]. In breast cancer, pharmacologic blockade of Yap through administration of curcumin induces oxidative stress damage in breast cancer and thus limits cell growth rate *in vitro* [63]. In septic cardiomyopathy, Yap deficiency activates mitochondrial stress through inhibiting ERK pathway, resulting into cardiomyocyte death in a manner dependent on mitochondria-initiated apoptotic pathway [64]. In cerebral hypoxia-reoxygenation injury, knockdown of Yap reduces gliocyte-mediated tissue regeneration through inhibiting the ROCK1/F-actin pathway [65].

Finally, we found that the F-actin/lamellipodium signaling is also modulated by Yap under hypoxic conditions. F-actin-mediated lamellipodium formation has been identified as a necessary step for cancer migration and invasion. We observed that lamellipodium degradation, partly due to F-actin transcriptional downregulation, was induced by hypoxia [66]. Interestingly, this effect could be enhanced by Yap knockdown, suggesting that Yap favors breast cancer mobilization under hypoxic stress. Similar to our finding, lamellipodium-related gastric cancer migration is also governed by Yap through the SIRT1-Mfn2 pathway [67]. In squamous cell carcinomas [68] and endometrial cancer [69], F-actin homeostasis is also sustained by Yap. Therefore, our results provide a novel insight into the molecular mechanism underlying breast cancer migration. Targeting the Yap/F-actin/lamellipodium pathway could be a promising approach to control breast metastasis.

## Figures and Tables

**Figure 1:** Yap knockdown induces breast cancer cell death and proliferation arrest under hypoxia stress. (a) MTT assay for cell viability in MCF-7 cells. siRNA against Yap (si-Yap) was transfected into cell before 24–48 hours hypoxia. (b) TUNEL staining was used to observe the cell apoptotic rate. siRNA against Yap (si-Yap) was transfected into cell before 24–48 hours hypoxia. (c) Caspase-3 activity was measured through ELISA. (d) qPCR was used to determine the efficiency of knockdown after si-Yap transfection. (e) CCK-8 assay was used to observe the cell proliferation capacity in MCF-7 cells under hypoxia. (f, g) qPCR assay was used to detect the transcription of VEGF and *p*21 in MCF-7 cells transfected with si-Yap. ^*∗*^*p* < 0.05.

**Figure 2:** Yap knockdown reduces mitochondrial function in hypoxia-treated breast cancer. (a) ATP production was measured through ELISA. (b, c) Mitochondrial membrane potential was determined in MCF-7 cells. siRNA against Yap (si-Yap) was transfected into cells before 24 hours hypoxia. (d, e) ROS production was detected in response to Yap knockdown. (f) Mitophagy activity was determined through the mt-Kemia assay. (g, h) qPCR assay was used to detect the transcription of Mfn2 and Opa1 in MCF-7 cells transfected with si-Yap. ^*∗*^*p* < 0.05.

**Figure 3:** Yap maintains mitochondrial homeostasis through activating HIF1 in MCF-7 cells under hypoxia. (a) The transcription of HIF1 was determined via qPCR in MCF-7 cells under hypoxia. (b) HIF1 expression was detected in response to Yap knockdown in the presence of hypoxia in MCF-7 cells. (c) ATP production was measured through ELISA. (d) ROS production was measured in response to Yap knockdown in the presence of hypoxia. ^*∗*^*p* < 0.05.

**Figure 4:** Overexpression of HIF1 abolishes Yap knockdown-mediated breast cancer cell death and proliferation arrest. (a) MTT assay for cell viability in MCF-7 cells. siRNA against Yap (si-Yap) was transfected into cells before 24 hours hypoxia. HIF1 adenovirus (ad-HIF1) was transfected into Yap-deleted MCF-7 cells before 24 hours hypoxia. (b) TUNEL staining was used to observe the cell apoptotic rate. (c) CCK-8 assay was used to observe the cell proliferation capacity in MCF-7 cells under hypoxia. (d, e) qPCR assay was used to detect the transcription of VEGF and *p*21 in MCF-7 cells transfected with si-Yap. ^*∗*^*p* < 0.05.

**Figure 5:** F-actin/lamellipodium signaling pathway is impaired by Yap knockdown under hypoxia. (a–c) Immunofluorescence for lamellipodium. The average length and number of lamellipodia was determined. siRNA against Yap (si-Yap) was transfected into cells before 24 hours hypoxia. HIF1 adenovirus (ad-HIF1) was transfected into Yap-deleted MCF-7 cells before 24 hours hypoxia. (d) qPCR was used to detect the alterations of F-actin in response to hypoxia, si-Yap transfection, and ad-HIF1 infection. (e) Transwell assay was used to observe the migratory response of MCF-7 cells. ^*∗*^*p* < 0.05.

## Data Availability

The datasets used and/or analyzed during the current study are available from the corresponding author on reasonable request.
